The article "Enterprise Operational Resilience with Digitalization Approach amid the COVID-19 Era: An Empirical Assessment" was published in 2022. Journal: J Environ Public Health.

# Enterprise Operational Resilience with Digitalization Approach amid the COVID-19 Era: An Empirical Assessment

**DOI:** 10.1155/2022/6274670

**Published:** 2022-10-28

**Authors:** Jinsheng (Jason) Zhu, Hui Zhang, Wenyong Feng

**Affiliations:** ^1^Belt and Road International School, Guilin Tourism University, Guilin 541006, Guangxi, China; ^2^Department of Tourism Management, Xinzhou Teachers University, Xinzhou 034000, Shan'Xi, China

## Abstract

The development of the COVID-19 pandemic has had a devastating impact on one Chinese city that has depended heavily on tourism, which is the core focus of the current study. This article uses phenomenological research methods in qualitative research to conduct semistructured and in-depth interviews with travel agency managers in China Highlights. Through the application of tourism resilience theory in the tourism crisis management domain, this article investigates the performance of China Highlights, a local tourism enterprise in Guilin, China, to restore the functioning and growth of the tourism industry in the postpandemic period. The results show that China's tourism industry is in the early stages of the fast growth stage of economic recovery, and tourism enterprises are faced with a significant challenge in determining how to make sound business choices during the pandemic and after the crisis has passed. It proposes that the tourism resilient theory can serve as a modern crisis management model to facilitate tourism enterprises to revive their performance in times of hardship.

## 1. Introduction

The income generated by domestic tourism in China in 2019 was around 5.73 trillion yuan, representing an increase of 11.7 per cent year-on-year [1–3]. As a result of the pandemic caused by COVID-19, domestic tourism ground to a halt within a short period, and the subsequent decline was considerable [4]. According to the calculation done by the China Tourism Academy for the year 2020, the two primary growth indices of domestic tourism revenue and domestic tourism population both indicated considerable declines in growth, with respective ranges of 18.6% to 29.9% and 13.9% to 19.5% [5]. In addition to this, the effect of the COVID-19 pandemic crisis on the revenue of domestic brigades was far more severe than the impact that SARS had [6, 7]. According to official figures from the Ministry of Culture and Tourism, international tourism revenue in 2019 was US $131.3 billion, up about 3.3 per cent year on year, with about 145 million inbound tourists, up about 2.9 per cent year on year. The China Tourism Research Institute has projected that the negative growth ratio of inbound tourism to international tourism revenue will be between 18.9% and 40.7% and between 21.9% and 44.5%, respectively [2]. The pandemic caused by COVID-19 has had a significant influence on the growth of the industries of culture and tourism all over the globe [8]. On the one hand, the tourist business has been hit hard by the effects of the COVID-19 pandemic, which has resulted in a significant decline in the sector's development trend. More than a 70 per cent to 90 per cent drop in both the overall number of visitors and the total consumption was seen between the year 2020 and 2021 [9]. Both the number of tourists coming into China and the country's overall spending have decreased by more than 90 per cent [10].

The article "Enterprise Operational Resilience with Digitalization Approach amid the COVID-19 Era: An Empirical Assessment" was published in 2022. Journal: J Environ Public Health.

Guilin was one of the first cities in China to establish its tourist industry, and as a result, a significant amount of the area economy's revenue comes from tourism. Statistics show that Guilin's tourist industry contributed over thirty to forty per cent of the overall GDP in 2017 [11, 12]. As a result, the tourist sector is an essential component in the continued growth of Guilin's economy. Guilin is a great example of a city that thrives off of tourism and may thus serve as a model for other cities across the world. The tourism sector in Guilin is a significant driver of economic growth and helps elevate people out of poverty [13, 14]. The COVID-19 outbreak has had a significant impact on the global economy and tourism sectors. The government established a series of countermeasures and strategies in order to mitigate the market, stabilize the monetary sector, and foster macroeconomic stability [15]. However, the development of the COVID-19 pandemic has had a devastating impact on one Chinese city that has depended heavily on tourism, which is the core focus of the current study.

It is anticipated that the recovery of the domestic tourist business would proceed at a slower rate, particularly considering that domestic tourism is still subject to stringent COVID-19 restrictions throughout China. It is crucial to research Chinese financial spillovers on other countries since China has been the first major country to rebound from the COVID-19 outbreak and the economic recovery of China served as a catalyst for expansion in all other countries [16]. Businesses that focus on cultural tourism are finding it difficult to go back to work and resume production [17]. Despite the fact that the findings of Wang and Su [18] lend credence to the idea that stringent quarantine procedures have the potential not only to shield the general population from the COVID-19 virus but also to have a beneficial effect on the surrounding natural ecosystem. These results may serve as a point of comparison for other nations as they evaluate the impact that COVID-19 has had on the environment. However, it will be very challenging for these businesses to go back to regular operations since they are dealing with obstacles such as municipal lockdowns and travel limitations from city to city. The pandemic caused by COVID-19 has left Guilin's tourist industries with two major research areas to investigate: how can tourist businesses strengthen their capacity to withstand potential dangers? Companies in the tourist industry that are in the early stages of the fast growth stage of economic recovery are confronted with a significant challenge: how to make appropriate business choices during the pandemic and in the postpandemic era? To answer these research questions, in-depth, semistructured interviews were conducted with managers at travel agencies in China using phenomenological research methodologies for this study. This article explores the efforts of China Highlights, a local tourist firm in Guilin, China, to revive the sector's operations and stimulate development in the wake of the pandemic by applying the tourism resilience theory to the tourism crisis management field. Based on these research efforts, it is clear that China's tourist sector is in the early stages of the rapid development period of economic recovery and that it will be a major problem for tourism firms to figure out how to make good business decisions during and after the pandemic. In times of crisis, it is suggested that the tourism resilient theory may be used as a model for effective crisis management, helping to restore the viability of the tourist industry. In the parts that follow, these issues are going to be discussed in an increasingly in-depth way.

The article "Enterprise Operational Resilience with Digitalization Approach amid the COVID-19 Era: An Empirical Assessment" was published in 2022. Journal: J Environ Public Health.

## 2. Literature Review

The concept of tourism resilience is used in this article for the management of tourist businesses during a time when such businesses are experiencing a crisis in the tourism industry [19, 20]. From a linguistic point of view, the word resilience originates from Latin, which means to revert to the initial condition [21]. The primary objective of the literature study is to get an understanding of the appropriate directives and procedures that travel industry operators have issued in the midst of a crisis [22, 23] and how tourism companies should achieve economic recovery after the crisis [24]. Among them are the capacity of travel businesses to effectively handle an emergency [19], and the ability of companies to transform traditional industries in times of crisis [25]. The idea of tourism crisis management [1, 26] is an essential theoretical basis for scientific prevention and management of large public health catastrophes, as well as an efficient reaction to these events. The early theoretical model [27, 28] and the fundamental theory of tourist disaster management [29] are some of the most important components in the field of tourism crisis management theory. These components can be modelled as reduction, readiness, response, and recovery, respectively [30, 31].

The article "Enterprise Operational Resilience with Digitalization Approach amid the COVID-19 Era: An Empirical Assessment" was published in 2022. Journal: J Environ Public Health.

Travel companies are affected by uncertain crises such as earthquakes and tsunamis, financial crises, politics, and crime [19, 32]. Numerous economic downturns have been a barrier to the growth of tourism-related businesses. It is possible to explain why the tourist sector is required to build crisis plans by positing that a crisis is most likely to have an impact on the growth of tourism enterprises. The capacity of a system to self-repair in the event that it is disrupted by either internal or external sources is referred to as its resilience [33]. Companies in the tourist industry that are in the early stages of the fast growth stage of economic recovery confront a significant challenge in determining how to make sound business choices during the pandemic and postpandemic eras. The management of tourist businesses should constantly strive to have a high level of crisis awareness at the forefront of their minds. The potential for industry change presents itself in the shape of the COVID-19 pandemic that is now affecting the tourist sector. It is imperative that small and medium-sized tourist businesses insist on the development of innovative products and services. This is because small and medium-sized tourism businesses have a greater capacity to tolerate risks than large-scale tourism businesses. At a macroscope, the construction of a tourist risk management system on a national scale has to be taken into consideration by the governmental guidelines pertaining to China's tourism risk management. At the microlevel, travel agencies should construct a crisis warning system in the case of large-scale public health crises, build a tourist service network system, and alter the business goal model of travel agencies.

In the same way that the term sustainability has been utilized by the academic community, the word elasticity has also been employed [34–36]. Elasticity is often used to describe an item that can return to its former shape or position after being bent, stretched, or otherwise deformed [37]. The description of the resilience idea echoes elasticity, which not only derives from the natural sciences and the flexibility applied to the social sciences, but it is also often used to characterize the capacity of communities to endure harsh situations. The first application of resilience theory in the tourist sector focuses on resilience and complex adaptive tourism systems [38, 39]. The capacity to strengthen tourist operations in the face of natural catastrophes and violent situations is resilience. The essential small and medium-sized tourist businesses are seen as relatively undeveloped, yet they indicate the growth of the entire tourism sector [40]. For instance, if you want to comprehend the resiliency of the whole tourist business after a natural catastrophe, you must focus on more than the recovery from economic losses. Greater emphasis should be placed on the recovery of supply chain services and associated businesses [41]. This approach is equally relevant to several communities and other economic activities unrelated to travel, although this book focuses on flexible applications in tourism.

The article "Enterprise Operational Resilience with Digitalization Approach amid the COVID-19 Era: An Empirical Assessment" was published in 2022. Journal: J Environ Public Health.

## 3. The Research Site, Problem Identification, and Research Questions

During the pandemic, the tourist sector will surely undergo a rearrangement and restructuring, which is also the industry's natural tendency toward high-quality development [42, 43]. How to capture the vein of tourism development during the pandemic and swiftly establish a new scenario after the pandemic has become a concern for tourism industry owners. Consequently, the current paper will concentrate on answering the following two research objectives: (1) how can effective efforts be taken to restore the functioning and growth of Guilin tourist businesses in the postpandemic period? (2) The postpandemic era's new tourist market supply dilemma. The following sections analyze the performance of a typical travel agency in Guilin in an effort to revive the local tourism market, meet the personalized needs of tourists, and improve the quality of tourism services. It is intended to investigate how Guilin city plans to optimize the tourism development environment, attract tourists for consumption, establish and implement the crisis plan, and restart and revitalize local tourism.

China's Guilin city in Guangxi Zhuang Autonomous Region was the primary focus of this study, especially in light of the COVID-19 outbreak. In the year 1998, China Highlights was established as an independent state-owned company [44]. It was one of the first tourist websites to be established on the Internet in China and was a forerunner in the development of the business model of inbound tailored tourism. In the past, this division of Guilin China International Travel Service Co., Ltd. was known as the e-commerce department. Its company and crew were split off from Guilin International Travel Service in August 2015, when the company was renamed. There are now 121 employees working for the company, many of which are natives of other nations such as the United Kingdom, Ireland, New Zealand, and other markets. Its primary focus is on catering to the needs of foreign tourists travelling around China by offering individualized assistance with trip planning and booking as well as travel greeting services. More than 40,000 travellers from outside of China use the company's travel services every year. Its websites are available in seven different languages, including English, German, Spanish, French, Japanese, Russian, and Italian. It is well-recognized that China Highlights puts an emphasis on quality first. The scope of the cooperation includes more than 300 outstanding multilingual contractual tour guides in more than 50 cities, including Beijing, Shanghai, and Xi'an, and they were the first to create a feedback form system for each tour guide as well as an annual tour guide assessment system. In addition to this, the company has established direct commercial partnerships with picturesque spots, hotels, and aviation agencies in significant cities all across the country. This was done to ensure that the best prices and the finest quality are supplied to customers. For international visitors to China, China Highlights, sometimes referred to as China Tour, is a company that plans itineraries and offers travel services around the country.

The article "Enterprise Operational Resilience with Digitalization Approach amid the COVID-19 Era: An Empirical Assessment" was published in 2022. Journal: J Environ Public Health.

As a result of the pandemic's continued spread around the globe, the travel advisory level for China will eventually be raised to its maximum level by numerous nations that are considered to be its sources. It is certain that the performance of the company would plummet dramatically over the next three years due to the pandemic that has been going on. At the same time, China Highlights forecasts that after the pandemic is eradicated, China Highlights will receive an increase in orders, particularly travel reservations for neighbouring countries and travel reservations for free travel. This forecast is based on the robust support that China Highlights has in the domestic segmented industry traffic, products, and brands. The burden that has been put on China Highlights' cash flow will be effectively relieved as a result of the wave of planned modest peaks that will be occurring. Consequently, while the situation is challenging, the overall operational risks faced by the organization are manageable. This indicates that it is anticipated that the company's business would decrease by fifty per cent but that the cash flow will be able to be sustained for between one and two years.

## 4. Research Methodology

This research adopts a qualitative research methodology [45–47]. When conducting qualitative research, the process of describing and explaining the interview transcript is referred to as the process of developing an abstract theory [48]. This is because this process involves the generation of a theory as well as the description and explanation of the theory. In order to conceive and enlarge the category, the major strategies entail open coding of the interview's verbatim transcript [49]. The subcategories are followed by the main axis coding [50, 51], which connects the categories and subcategories along the straight line of attributes and orientations. The selected translation codes will be subject to unifying and refining the theory, organising it by a core concept, and outlining the theoretical framework. Furthermore, it proceeded to the next step of refining the theory, trimming redundant concepts, making up for under-developed categories, and so on. These will be followed by process coding, and we conduct a test of the entire coding process to develop a temporary theory. Thus, this article uses phenomenological research methods in qualitative research to conduct semistructured and in-depth interviews with travel agency managers in China Highlights. The subcategories come to the main axis coding, which joins the categories and subcategories along the linear progression of the orientations and qualities. In addition, it moved on to the following stage, which consisted of refining the theory, eliminating unnecessary notions, and filling in gaps left by underdeveloped categories.

The article "Enterprise Operational Resilience with Digitalization Approach amid the COVID-19 Era: An Empirical Assessment" was published in 2022. Journal: J Environ Public Health.

The following is a summary of the interview: (1) would you be willing to discuss the impact the pandemic has had on your present place of employment? (2) What kinds of challenges and obstacles does the organization face in the tasks related to administration? (3) In the event that a COVID-19 pandemic occurs, what should be done to address and resolve any issues that arise? The objective of this study, as well as its relevance, techniques, and substance, are all sufficiently informed to the respondents before the actual interview in the year 2020 and 2021. In order to ensure compliance with the concept of secrecy, the interviews were taped and made a part of a procedure only after receiving informed permission from the participants. During the course of the interview, the authors paid careful attention to observing and recording changes in the interviewee's expression, speaking speed, and intonation. In addition, the authors utilized interview techniques such as rhetorical inquiry, follow-up, repetition, summary, and response in order to obtain the views and feelings that were most genuine. Interviews with each manager typically last between 25 and 40 minutes. The authors were ultimately able to abstract the results by doing a methodical study of the original data and progressively summarizing it into abstract thinking. This allowed the authors to achieve conclusions that were founded on empirical collections and facts. After that, grounded analysis was used to interconnect theoretical research with empirical research, which is a frequent practice in scientific research.

The article "Enterprise Operational Resilience with Digitalization Approach amid the COVID-19 Era: An Empirical Assessment" was published in 2022. Journal: J Environ Public Health.

### 4.1. Open Coding

During the stage of open synthesis, this study will assess and compare the original data that were obtained from the interview and will also summarize the ideas and categories [52]. Throughout the whole, open-coding process, an attitude of objectivity was consistently maintained. In the original materials, all of the gathered films, notes from the interviews, researchers' thoughts and observations, the original questionnaires, and research memoranda are brought together. The project carried out open coding on the original sentences obtained from the interviews, and as a result, it obtained a total of 386 original sentences and the initial concepts that corresponded to them. This was performed with an orientation toward the influencing factors of the pandemic recovery strategy. The authors examined and improved the ideas of the interviewees, combined the concepts that were overlapping, got rid of the initial concepts that occurred less often (fewer than three times), and eventually accomplished conceptual classification, thus narrowing down to 12 fundamental categories.

### 4.2. Axial Coding

In order to discover the interrelationships between ideas and to incorporate higher-level categories by conducting more research and analysis on open coding, the goal of axial coding is to determine the interrelationships between concepts. This study group has outlined four primary categories of variables impacting the recovery of tourist firms under the effect of the pandemic. Their conclusions are based on the interrelationships that exist between the various categories of factors. These four fundamental categories evolve into the key ideas that underpin the integration of the rest of the categories. The axial coding was followed by an extension of the primary themes derived from the phenomena that were noticed in the study.

### 4.3. Selective Coding

During the step of selective coding, all of the specified idea categories are subjected to the integration and condensing process, which ultimately results in the formation of four primary categories. At this step, the primary task is to integrate and enhance the conceptual categories that have been identified, with the end goal of improving the core category.

### 4.4. Saturation Test

The process of analysis will continue until the researchers have reached a point of saturation; when they have reached this point, there will be no new ideas which have emerged from the data that has been gathered. Instead, the researchers saw a significant recurrence of the individuals' statements that were either explicitly articulated or previously observed. As a result, the findings of this study have shown the value of saturation and accomplished a level of high validity and trustworthiness.

The article "Enterprise Operational Resilience with Digitalization Approach amid the COVID-19 Era: An Empirical Assessment" was published in 2022. Journal: J Environ Public Health.

## 5. Research Findings and Strategic Analysis

### 5.1. National Governance Countermeasures Are in Favour of Tourism Resilience and Enterprise Recovery

Businesses are able to adapt and make it through the crisis thanks to changes in government policy [53–55]. Since the beginning of the COVID-19 outbreak, the central state as well as the cultural and tourism authorities have actively responded and implemented measures to assist in the bailout of tourism companies [56]. These actions include the reimbursement of travel agency guarantee money, the strengthening of the protection of tour guides' labour rights, and the issuance of guidelines for the return of employment and production. In addition, local governments have implemented measures to increase cultural and tourism consumption, such as free admission policies for medical staff, the issuance of travel vouchers, the establishment of cultural and tourism industry relief funds, and the introduction of online tourism training courses to assist travel enterprises in overcoming obstacles [57]. These policies and projects are intended to encourage more people to participate in cultural and tourism activities. These guidelines and training programs are intended to assist firms in the travel industry in overcoming obstacles. These steps not only reduce the strain that is being placed on organizations and businesses related to tourism in the near term, but they also encourage the recovery and expansion of the tourist sector, as well as its transformation and upgrading [58, 59]. Despite the fact that the COVID-19 pandemic has had an impact on travel throughout the world, China's internal tourism has recovered partially. Although the pandemic has had a chilling effect on overseas trips, domestic tourism in China has shown some signs of improvement. The fact that Chinese visitors may now enjoy duty-free discounts on several goods, including cosmetics and electronic items, without having to travel outside of China is another factor that is contributing to the resurgence of China's domestic tourism sector. Even though the COVID-19 pandemic has led to a decrease in the travel demand and even though the foreign tourist sector is currently in a state of decline, it is anticipated that tourism and shopping inside China would see a surge in tourist activity, as Caballini et al. termed this as tourist mobility [60]. The interview that was conducted by China Highlights has also shown their optimistic attitudes concerning the devastating consequences of the pandemic:

*“From an industry perspective, I think China Highlights is characterized by online e-commerce, inbound tourism, and customized grouping, and it is also a type of small and medium travel agency. Therefore, compared with the entire industry, the losses suffered are moderate to low, and the recovery period is medium to long. Once we have overcome the immediate difficulties, recovery and growth should come at the same time* (Interview with one of the board members in the China Highlights).”

The article "Enterprise Operational Resilience with Digitalization Approach amid the COVID-19 Era: An Empirical Assessment" was published in 2022. Journal: J Environ Public Health.

These comments demonstrate that tourism resilience serves as the critical theory to understand how national policies, tourism enterprises, and destination-oriented individuals could strive for active responding and adaptive survival while facing global changes and market adversities [61–63]. This is particularly important now that COVID-19 has been wild-spread throughout the global tourism industry. On the one hand, concepts of resilience such as eco-systematic resilience are easily ingrained in academic kinds of literature [64]. On the other hand, organizational enterprises such as the national-level administrative board and the business that we are researching, China Highlights needs to also take into consideration these systematic mindsets. To conclude this section, the authors reiterate that the eco-systematic resilience thoughts are a wide-ranging, multifaceted, and well-organized cluster of mindsets [65, 66].

### 5.2. Digitalization as a Coping Strategy of China Highlights Seen from the Perspective of the Tourism Enterprises

Tourism businesses must significantly change their internal and external resilience to withstand the crisis's consequences [67]. To understand the current situation of the resumption of work and production of tourism companies and the public's tourism consumption awareness, the authors interviewed the general manager of the China Highlights, covering the ideas such as digital, networking, socialising, and interactive tourism products production methods for the sustainable development of the tourism industry and tourism enterprises. One of the managers concludes as follows:

*“The tourism industry is undoubtedly affected by the impact of COVID-19. However, according to the characteristics of the entire industry, the degree of impact and recovery cycle of different companies are different. In the long run, tourism is still rare in the “sustainable sunrise industry,” which means that recovery and growth often occur simultaneously. Our strategies to cope with the SARS impact in 2003 were a good example. Taking into account the breadth and depth of the SARS impact that year, it is generally believed that it will take about 2 years for the entire industry to recover. China Highlights' guiding response measures during the pandemic include is to cover the money bag and increasing capital withdrawal, seeking low-cost loans to increase cash reserves* (Interviewed one of the managers in China Highlights, in which he expressed his positive vision on the overall recovery of the tourism industry. The interview was conducted in Chinese and translated into English in November 2020).”

The article "Enterprise Operational Resilience with Digitalization Approach amid the COVID-19 Era: An Empirical Assessment" was published in 2022. Journal: J Environ Public Health.

Tourism is a sensitive but not fragile industry. Sensitivity here means that any visible or potential natural disasters, geopolitics, international relations, the economy of the source country, public safety, and pandemics will be converted into cancellation in the industry. Every outbreak of similar incidents is the pain of the entire industry. Not fragile here means that travel is an advanced spiritual pursuit that cannot be given up. Demand will be temporarily suppressed, but it will never disappear. Once the visible crisis is eliminated, travel needs will be released. As the pandemic continues to spread overseas, and many source countries (the United States, Australia, and others) will raise the warning level for Chinese travel to the highest level. Even if it is confident that the business would start to bounce back by the end of 2022, a precipitous decrease in performance over the past three consecutive years amid the COVID-19 pandemic is inevitable. Nevertheless, if the firm responds vigorously and increases its recovery investments, the yearly performance of the following year in 2022 is predicted to return to between 55 and 65 per cent of its original level in 2019 year-over-year. If the crisis worsens or the situation necessitates prudence, it is projected that the performance of China Highlights would witness another significant decline in the upcoming years.

Another strategy for the survival of tourism enterprises under the impact of COVID-19 lies in its information technology advancement and operation [68, 69]. Digital cultural tourism such as online video, online audio, online education, and payment for knowledge presents more obvious development advantages [69]. These fundamental countermeasures will expedite the progression of the tourist business to the next stage, which will include digitization, intelligence, and socialization [70]. In the face of the gradual rejuvenation of the market after the pandemic, challenges and development opportunities are faced in the three aspects of product upgrades, marketing upgrades, and industrial intelligence. According to the interview, because of the protracted length of the home pandemic, the majority of firms and industries have been impacted, and the income of some individuals has decreased or even lost, which has exacerbated psychological torture over the pandemic. The interview indicates that the pandemic has placed the tourism business in a sensible cooling-off period. The advent of the pandemic will allow businesses with weak core capabilities to withdraw from the market first, hence strengthening the tourism industry's emphasis on resilience. The pandemic will also generate new business forms and models, so changing people's consuming conceptions and patterns of consumption. A participant in the interviews in this research expressed these words:

*“We plan to respond to this period of restructuring in the industry more aggressively by relying on large cash flow as well as leading market and brand advantages. The occurrence of a major catastrophe will always result in the need for fresh adjustments or the acceleration of the process of incrementally improving business models. The COVID-19 pandemic has given birth to new tourism business formats and new service models. Some examples of these include real-name registration, a sharp drop in offline passenger flow, and the digital force of intelligent management in scenic spots. These new business formats and service models were made possible thanks to the active exploration and joint efforts of the tourism industry. Businesses are competing for beachfront property in what has become known as the “New World” of tourism: online tourism and cross-border sales. “Contactless service” results in “smart unmanned hotels,” which helps promote the shift that the tourism industry has to make to recapture customers* (Interviewed with one of the most senior managers working on China Highlights. The interview was carried out in Chinese, and a translation into English is scheduled to take place in November 2020).”

The article "Enterprise Operational Resilience with Digitalization Approach amid the COVID-19 Era: An Empirical Assessment" was published in 2022. Journal: J Environ Public Health.

Adopting an adaptive strategy while facing the pandemic, China's tourism industry has actively carried out the features of internal circulation, including promoting the transformation of digitalization [71], upgrading software and hardware facilities in scenic spots, strengthening staff training, and improving the overall service level of scenic spots. Scenic spots cooperate with Internet companies to carry out live broadcast activities (also termed virtual tourism during the pandemic era) [72, 73] and actively formulate pandemic prevention. Tourism companies strive to protect the rights and interests of consumers, and they have launched tourism revival plans to spare no effort to restore energy for the tourism industry affected by the pandemic.

The tourism industry is an industry that is sensitive to external factors and is often exposed to multiple risks, but it is also an industry with great resilience and vitality. Most of the precedential studies show that the tourism industry has entered a stage of development of a more mature industry and has good endogenous growth momentum [74–76]. After the pandemic is ended, there will be an upsurge in the demand for national consumer goods, which will lead to a gradual release of the demand that had been repressed for tourism. This would usher in a period of boom for the tourist sector. We need to expand brand coverage while expanding market share and create optimal preparations for the industry restructuring's accelerated resurgence.

### 5.3. Individual-Level Tourism Resilience for All Lines of Staff in the Tourism Industry

The crisis-resistance capacity of tourism practitioners may be bolstered through legislative assistance for tourist businesses [77, 78]. The first effect of COVID-19 on individual employees in the tourist business is a decline in revenue. Individual lives will be impacted by the pandemic to varying degrees, depending on how well the tourist industry rebounds. Everyone is under pressure from mortgages, auto loans, and rent, as well as family assistance, children's education, and parents' pension expenses. In addition, the compensation of some workers seems to be the sole revenue source for some families. More importantly, each individual may still face the pressure of rising prices due to material shortages. Despite that the company reduces welfare expenses and advertising expenditures and suspends investment in marginal tentative businesses, the company is still facing a hardship situation. It is precisely because of the company's social responsibility that management must endeavour to provide additional options for tourist employees to generate revenue within the organization. In the interview, the interviewees expressed the adaptive strategies among the front-line officers:

*“China is the country most affected by COVID-19 in the first stage of this pandemic. Therefore, our jobs and positions have been integrated and adjusted. When orders drop to almost zero and the travel teams are faced with full cancellations, we will inevitably have many positions that are not saturated with the original work. The same is true for market personnel. To increase the input-output ratio, our focus must also be adjusted. We need to conduct training, self-improvement and re-organize the work process, and the system construction team. We need to improve our abilities in a real sense: consultants need to design innovative tourism products; the product marketing department needs to produce novel information for the market; information IT managers need to renovate our digital working platforms; what's more, tour guides service need to upgrade the training efforts to better facilitate the market needs* (Interview with the strategic manager in China Highlights in November 2020).”

The article "Enterprise Operational Resilience with Digitalization Approach amid the COVID-19 Era: An Empirical Assessment" was published in 2022. Journal: J Environ Public Health.

At present, almost all companies in the country that can support remote work are looking for full-process office solutions. The company's management began to work remotely, greatly improving communication efficiency, concentration, attendance management, and other problems. Collaborative office in different places around the world has become a possible option. The tourism industry also needs to think further: what iteration of our management model needs to be done? What kind of talent strategy should the tourism industry need?

## 6. Discussion and Conclusion

According to the interview data, owing to the extended duration of the domestic pandemic, the majority of firms and industries have been impacted, and the income of some individuals has decreased or even disappeared, which has exacerbated the psychological terror surrounding the disease. Tourist resilience is essential for comprehending how national policies, tourism businesses, and destination-oriented people can combat global change and market difficulties, particularly while COVID-19 is raging. Given the huge uncertainty of the COVID-19 pandemic, it is difficult to make accurate predictions in the short term. However, the widespread effects of the pandemic have increased macro-level unpredictability. It coincides with the breakthrough in the transformation and upgrading of China's tourism industry, which has increased the most variables of industry development.

Tourism decision-making is inseparable from the interesting relationship between the government, tourism companies, tourism practitioners, and all related stakeholders [79]. Tourism companies are responsible for the interesting relationship between the government and tourists, particularly during crises [80]. Sudden major public safety and health incidents have paralyzed the national tourism industry. Millions of orders were cancelled, hotels, restaurants, and tourist theme parks were closed, and the transportation industry ceased services. Tourism is China's third-largest industry midstream economic pillar, connecting thousands of side-chain industries. The future of tourism development in the postpandemic era has become a hot topic at the moment, deriving emerging tourism methods such as medical tourism, green health tourism, and rural eco-tourism. People pay more attention to their health and are no longer satisfied with their simple eating, wearing, housing, and transportation in the past. This level of demand is a huge change for practitioners in the tourism industry, and tourism practitioners need to provide services that are more in line with current needs. With the development of the Internet, the form of tourism is changing. When the pandemic comes, to satisfy tourists who can enjoy the beautiful scenery without leaving home, the same scenic spots must provide corresponding cloud viewing services. The postpandemic era is a huge era of innovation. Constantly learning new concepts, updating traditional concepts, and integrating existing new models are new challenges facing the development of the tourism industry.

The article "Enterprise Operational Resilience with Digitalization Approach amid the COVID-19 Era: An Empirical Assessment" was published in 2022. Journal: J Environ Public Health.

In this paper, we evaluate the performance of a local tourist business called China Highlights by using the tourism resilience theory inside the tourism crisis management arena. This article provides a summary of the three layers of management, specifically the policy-enterprise-individual eco-systematic matrix, in order to investigate the policy analysis on the national level, the operational adjustment of the company, the enterprise survival strategies under the pandemic, and the representative changes that occurred in individual-level staff. It contends that the tourist resilience theory has the potential to function as a contemporary model for crisis management, with the aim of assisting tourism businesses in reviving their performance in the face of adversity. In particular, the countermeasures and regulations that have a national scope contribute to the creation of a macroscope that bounces the outside environment for the tourist business. Enterprises in the tourism industry people need to actively take action that is both flexible and adaptable in order to accommodate themselves to the pandemic issue on an internal and external level. The working staff in these tourism businesses needs to take a strategy of retrenchment in order to control the expenses of the company and to increase their productive capacity during the affected daily routine in the pandemic era, while waiting for the opportunity to rejuvenate in the era after the pandemic.

The pandemic offers a useful opportunity for the tourist business to take a breather and regroup during this strategic lull. The emergence of the pandemic will make it possible for certain businesses that lack strong fundamental skills to depart the market first, which will lead to an even greater concentration of buyers in the tourist sector. The pandemic will also give rise to certain new business forms and models, which will in turn reshape people's notions about consumption as well as their behaviors around consuming. Companies in the tourist sector need to get a better understanding of the external development environment and trends, improve the clarity of their thinking, and locate the appropriate course of action in order to facilitate the speedy recovery of the tourism business after the pandemic has ended. In spite of the fact that all of the tourist industry's stakeholder lines are being negatively impacted by the pandemic caused by COVID-19, they are simultaneously incubating prospects for changes in the market as a result of this pandemic.

The article "Enterprise Operational Resilience with Digitalization Approach amid the COVID-19 Era: An Empirical Assessment" was published in 2022. Journal: J Environ Public Health.

The following are some of the limitations of this particular paper: to begin, the scope of this investigation is limited to a single tourist business as its case study. The objections to the results were restricted as a result of the breadth of the research aim. Second, the research technique that was used in this study has a long way to go before it is perfect; it has to have a greater focus on statistical analysis and a quantitative strategy. The authors of this article have high hopes that it will, in the future, inspire more Chinese tourism businesses to bravely investigate the pandemic storm and become pioneers in this industry. Additional studies should also concentrate on the cultural and marketing aspects of the case study.

## Data Availability

The authors confirm that the data supporting the findings of this study are available within the article.

## Additional Points

*Highlights*. (1) The COVID-19 pandemic has caused severe impacts on global economic, political, and socio-cultural systems, especially the tourism sector. (2) Tourism enterprises, as main players in tourism development, are facing critical moments. (3) A national-level administrative agency, tourism companies, and the front-line individual staff should jointly be united to combat the COVID-19 pandemic.
